# Real life triplet FIr/FOx chemotherapy in first-line metastatic pancreatic ductal adenocarcinoma patients: recommended schedule for expected activity and safety and phase II study

**DOI:** 10.18632/oncotarget.25870

**Published:** 2018-08-07

**Authors:** Gemma Bruera, Silvia Massacese, Stefania Candria, Antonio Galvano, Rosa Manetta, Aldo Victor Giordano, Sergio Carducci, Alessandra Di Sibio, Eugenio Ciacco, Antonio Russo, Enrico Ricevuto, on behalf of Oncology Network ASL1 Abruzzo, Italy

**Affiliations:** ^1^ Oncology Territorial Care Unit, S. Salvatore Hospital, Oncology Network ASL1 Abruzzo, University of L’Aquila, L’Aquila, Italy; ^2^ Department of Biotechnological and Applied Clinical Sciences, University of L’Aquila, L’Aquila, Italy; ^3^ Pharmacy Unit, S. Salvatore Hospital, Oncology Network ASL1 Abruzzo, L’Aquila, Italy; ^4^ Medical Oncology Unit, Department of Surgical, Oncological and Stomatological Sciences, University of Palermo, Palermo, Italy; ^5^ Radiology Unit, S. Salvatore Hospital, Oncology Network ASL1 Abruzzo, L’Aquila, Italy

**Keywords:** FIr/FOx, first-line, metastatic pancreatic ductal adenocarcinoma, phase II study, triplet chemotherapy

## Abstract

**Background:**

Gemcitabine/nab-paclitaxel and FOLFIRINOX demonstrated significantly increased survival compared with gemcitabine in metastatic pancreatic ductal adenocarcinoma (PDAC): objective response rate (ORR) 23 and 31.6%, progression-free survival (PFS) 5.5 and 6.4 months, overall survival (OS) 8.7 and 11.1 months. Present phase II study evaluated recommended first-line triplet FIr/FOx schedule.

**Methods:**

Simon two-step design: p_0_10%, p_1_30%, power 80%, α5%, β20%. Projected ORR: I step, 1/10; II 5/29. Schedule: 12h-timed-flat-infusion/5-fluorouracil 750-800-900 mg/m^2^ d1-2,8-9,15-16,22-23; irinotecan 120-140-160 mg/m^2^ d1,15; oxaliplatin 70-80 mg/m^2^ d8,22; every 4 weeks, according to clinical parameters (age, comorbidities, performance status (PS), liver function). Activity and efficacy were evaluated, and compared using log-rank; limiting toxicity syndromes (LTS), using chi-square.

**Results:**

Twenty-nine consecutive patients were enrolled, according to primary/intermediate/secondary Cumulative Illness Rating Scale (CIRS). Median age 62; elderly 13 (44.7%); PS2 3 (10.4%), secondary CIRS 5 (17.2%). Primary endpoint was met: ORR 53% (7/13 patients) as-treated, 50% intent-to-treat. Cumulative G3-4 toxicities: diarrhea 17%, asthenia 14%, hypertransaminasemy 7%, mucositis 7%, vomiting 3%, anemia 3%, thrombocytopenia 3%. LTS were 27.5% overall, 38.4% in elderly. At 3 months median follow-up, PFS 4 months, OS 11 months. PS2 patients showed significantly worse OS (*P* 0.022).

**Conclusion:**

Intensive first-line triplet FIr/FOx is tolerable at modulated doses, and confirms high activity/efficacy in metastatic PDAC. Patients’ careful selection, and exclusion of PS2, can maintain safety profile and efficient dose intensity.

## INTRODUCTION

Metastatic pancreatic ductal adenocarcinoma (PDAC) is a lethal disease with approximately 6 months median overall survival (OS) [1–3]. In the clinical evolution of metastatic PDAC, different combination treatment options have been evaluated, in order to increase clinical outcome. Gemcitabine was the only approved single agent, with median OS 5.7 months and 1-year OS rate 20% [1]. Gemcitabine 1000 mg/m^2^, administered over 30 minutes, weekly for 3 weeks every 28 days, was considered standard treatment schedule. Fixed-dose rate gemcitabine (10 mg/m^2^/minute) maximized intracellular concentrations of the phosphorylated active forms of gemcitabine, and may substitute standard infusion over 30 minutes [4, 5].

Even if phase III studies proposing gemcitabine-based associations failed to improve OS [6–16], excepting with erlotinib, a recent meta-analysis demonstrated that they achieved OS benefit in patients with good performance status (PS) [17]. Doublet gemcitabine-based associations with different drugs (cisplatin, oxaliplatin, fluoropyrimidine) reported objective response rate (ORR) ranging between 6.9-26.8%, progression-free survival (PFS) 2.7-6.0 months, OS 5.7-9.0 months, but failed to significantly increase OS [6–11, 13, 15]: gemcitabine plus oxaliplatin (OXP) increased ORR, PFS and clinical benefit, with no OS benefit, as reported with fixed-dose rate gemcitabine and OXP; capecitabine increased ORR and PFS, with a trend toward increased OS. Patients with PS 0-1 have shown a favorable or potentially favorable impact of gemcitabine-based doublets on PFS or OS. Gemcitabine combinations with targeted agents (bevacizumab, cetuximab) did not improved OS (5.8 and 8.8 months, respectively) [18–20]. The EGFR tyrosine kinase inhibitor erlotinib added to gemcitabine significantly improved OS compared to gemcitabine alone: median OS 6.24 months and 1-year OS rate 23%, with a significantly improved PFS, 3.75 months. More, bevacizumab addiction to this doublet chemotherapy significantly increased PFS 4.6 months, but not OS (7.1 months) [21]. Gemcitabine plus a platinum agent (i.e. cisplatin or OXP) could be also considered in patients with hereditary risk factors (*BRCA* 2 or *PALB* mutations).

The association of nab-paclitaxel to gemcitabine reported highest clinical benefit in patients with PDAC, and significantly raised up OS 8.7 months, PFS 5.5 months, and ORR 23%, compared with gemcitabine alone [22, 23]. Intensive triplet FOLFIRINOX regimen significantly prolonged OS up to 11.1 months, PFS up to 6.4 months, ORR 31.6%, compared to gemcitabine arm [24].

The most relevant issue limiting the feasibility of addition of more drugs in a chemotherapy combination is the proper design of the schedule assuring the balance between tolerability for individual patients and effective received dose intensity (DI) of each drug in order to obtain the expected efficacy of the combination. Intensive regimens based on triplet chemotherapy in MCRC, and FOLFIRINOX regimen in metastatic PDAC, frequently required proper clinical management of toxicity and treatment modulations due to moderate/severe toxicities [24, 25].

Over the last 10 years, we developed triplet chemotherapy regimen according to FIr/FOx schedule, characterized by 12-hour (10^PM^ to 10^AM^) timed-flat-infusion (TFI) 5-FU (TFI/5-FU), without leucovorin, associated to irinotecan (CPT-11) and OXP, according to a weekly alternating schedule, also added to bevacizumab [26, 27]. FIr/FOx showed efficacy equivalent to other triplet schedules, such as FOLFOXIRI [28, 29], with a good tolerability profile [30, 31], as first-line treatment of metastatic colorectal cancer (MCRC) patients, with increased received 5-FU DI and lower rate of grade 3-4 neutropenia. Intensive triplet chemotherapy plus bevacizumab, according to FIr-B/FOx schedule, was equivalently safe and feasible in young-elderly patients, selected by favourable PS, and comorbidity status. The evaluation of limiting toxicity syndromes (LTS), multiple site (LTS-ms) or single site (LTS-ss), represented an innovative indicator of toxicity of the individual patient [32, 33]. More, pharmacogenomic biomarkers of 5-FU, CPT-11 and/or OXP metabolism, could be evaluated to predict gastrointestinal toxicity in individual patients [34–36].

To further improve efficacy/tolerability ratio of triplet chemotherapy regimens in metastatic PDAC patients, the present phase II study proposes first-line FIr/FOx association [26, 27] in clinical practice.

## RESULTS

### Patient demographics

From February 2011 to September 2016, 29 consecutive, unselected patients were enrolled (Table 1): Male/Female ratio, 15/14; median age, 62 years; 10 (34.4%) young-elderly (yE) (≥65 <75 years), 3 (10.3%) old-elderly (oE) patients (≥75 years); World Health Organization (WHO) PS 0, 1, and 2, 16, 10, and 3 patients; Cumulative Illness Rating Scale (CIRS) [37] primary, intermediate, and secondary, in 10, 14, and 5 patients; metastatic disease metachronous in 2 (6.8%) patients, synchronous in 27 (93.1%) patients. Clinical diagnosis of PDAC was performed in 3 (10.3%) patients, hystological/cytological in 26 (89.6%) patients; these 3 patients, with typical clinical/laboratory presentation, and abnormal CA19.9 increase, did not underwent biopsy due to clinical features, poor PS, abnormal liver functional test. Primary tumor location was: head 17 (58.6%) patients, body 7 (24.1%), tail 5 (17.2%).

**Table 1:** Patients’ features

	Total N. (%)
No. of patients	29
Sex	
Male/Female	15/14
Age, years	
median	62
range	48-76
≥ 65 <75 years	10 (34.4)
≥ 75 years	3 (10.3)
WHO Performance Status	
0	16 (55.1)
1	10 (34.4)
2	3 (10.3)
Cumulative Illness Rating Scale (CIRS)	
primary	10 (34)
intermediate	14 (48.2)
secondary	5 (17.2)
Metastatic disease	
metachronous	2 (6.8)
synchronous	27 (93.1)
Diagnosis	
clinical	3 (10.3)
hystological/cytological	26 (89.6)
Primary tumor	
head	17 (58.6)
body	7 (24.1)
tail	5 (17.2)
Sites of metastases	
liver	18 (62)
lung	2 (6.8)
lymph nodes	22 (75.8)
local	2 (6.8)
cutaneous/subcutaneous tissue	1 (3.4)
peritoneal carcinomatosis	12 (41.3)
bone	2 (6.8)
No. of involved sites	
1	2 (6.8)
≥2	27 (93.1)
Single metastatic sites	
liver	-
lung	-
lymph nodes	2 (6.8)
local	-
peritoneal carcinomatosis	-
bone	-
Liver metastases	
single	1 (3.4)
multiple	17 (58.6)
Previous adjuvant chemotherapy:	1 (3.4)
gemcitabine	1 (3.4)
Previous radiotherapy:	1 (3.4)
Radiotherapy alone	-
Radiotherapy + chemotherapy (5-Fluorouracil c.i.)	-
Radiotherapy + chemotherapy (Capecitabine)	1 (3.4)

Abbreviations: WHO, World Health Organization; c.i., continous infusion.

Metastatic sites: liver 18 patients (62%), lung 2 (6.8%), lymph nodes 22 (75.8%), local recurrence 2 (6.8%), cutaneous/subcutaneous tissue 1 (3.4%), peritoneal carcinomatosis 12 (41.3%), bone 2 (6.8%). Metastatic site was single in 2 patients (6.8%), multiple in 27 (93.1%). Single metastatic sites: lymph nodes 2 patients (6.8%). Liver metastases were single in 1 patient (3.4%), multiple in 17 (58.6%).

Five patients underwent surgery of primary pancreatic tumor. One patient received adjuvant gemcitabine, 1 patient underwent radiotherapy associated with capecitabine.

Baseline CA19.9 measurement was normal in 3 patients, elevated in 26.

### Activity and efficacy

In the first step, according to two-steps Simon’s design [38], assuming as minimal interesting activity an ORR 10% (1 OR among 10 enrolled patients), OR were 3 out of 10 enrolled patients, ORR 30% in the intent-to-treat (ITT) analysis, and 5 out of 10 evaluable patients, ORR 50% in the as-treated analysis.

The phase II study was performed among the projected 29 patients. In the intent-to-treat analysis, 14 patients were evaluable, 13 patients did not received at least 3 cycles of treatments, and 2 patients were on-treatment at data cut-off. OR were 7 out of 14 patients, ORR 50% (α 0.05, CI ± 27) (Table 2): 5 objective partial responses (35.7%), 2 complete responses (14.2%); 3 stable disease (21.4%); 4 progressive disease (28.5%). Disease control rate was 71.4% (α 0.05, CI ± 24). In the as-treated analysis, 13 patients who received at least three cycles of treatment as planned were evaluable for activity (1 patient was evaluated after 2 cycles). OR were 7 out of 13 patients, ORR 53% (α 0.05, CI ± 27): 5 partial responses (38.4%), 2 complete responses (15.3%); 3 stable disease (23%); 3 progressive disease (23%). Disease control rate was 76.9% (α 0.05, CI ± 23).

**Table 2:** Activity and efficacy data

	Intent-to-treat Analysis		As-treated Analysis	
	No	%	No	%
**Enrolled patients**	29	100	29	100
**Evaluable patients**	14	48.2	13	44.8
**Objective Response**	7	50 (CI ± 27)	7	53 (CI ± 27)
Partial Response	5	35.7	5	38.4
Complete Response	2	14.2	2	15.3
**Stable Disease**	3	21.4	3	23
**Progressive Disease**	4	28.5	3	23
**Median Progression-free Survival, months**	4	89.6		
Range	0-21			
Progression events	26			
**Median Overall Survival, months**	11	82.7		
Range	0-33			
Deaths	24			

At median follow-up of 3 months (Figure 1), median PFS was 4 months (0-21): 26 events occurred and 3 patients (10.3%) were progression-free. Median OS was 11 months (0-33): 24 events occurred and 5 patients (17.2%) were alive. Among 13 yE/oE patients, median PFS was 4 months (1-21), median OS 5 months (1-33). PFS and OS were not significantly worse in elderly compared to non-elderly patients (*P* = 0.360 and 0.235, respectively) (Figure 2). Among the 16 patients treated with full standard dose, median PFS was 4 months (0-21), median OS 11 months (1-29+); among 13 patients treated with modulated doses due to age, comorbidities, PS, and/or abnormal liver function, PFS was 3 months (0-13), median OS 12 months (0-33). PFS and OS were not significantly worse in patients treated with reduced/modulated drugs doses compared to patients treated with full standard doses (*P* = 0.380 and 0.749, respectively) (Figure 2). Among the 3 PS 2 patients, median PFS was 1 month (1-3), median OS 1 month (1-3); among 26 PS 0-1 patients, median PFS was 4 months (0-21), median OS 12 months (0-33). OS was significantly worse in PS 2 compared with 0-1 patients (*P* = 0.022); PFS was not significantly different (*P* = 0.078) (Figure 2).

**Figure 1:** Kaplan-Meier survival estimates Overall enrolled patients; **(A)** progression-free survival; **(B)** overall survival.

**Figure 2:** Kaplan-Meier survival estimates 1, Elderly compared to non-elderly patients; 2, patients treated with standard dose compared to patients treated with modulated doses; 3, performance status 2 compared to 0-1 patients; 4, head compared to other tumor location; 5, liver metastases compared with other metastatic site; **(A)** progression-free survival; **(B)** overall survival.

Among the 17 patients with head tumor location, median PFS was 4 months (0-13), median OS 11 months (0-33); among 12 patients with other than head pancreatic tumor locations, median PFS was 2 months (0-21), median OS 3 months (0-25). PFS and OS were not significantly different (*P* = 0.896), even if OS was trendy worse in patients with other than head pancreatic tumor location (Figure 2). Among the 18 patients with liver metastases, median PFS was 3 months (0-21), median OS 5 months (0-33); among 11 patients with other metastatic sites, median PFS was 4 months (0-12), median OS 11 months (0-29+). PFS and OS were not significantly different (*P* = 0.601, and 0.869, respectively), even if OS was trendy worse in patients with liver metastases (Figure 2).

Ten patients (34.4%) received, at least, a second line treatment: FIr/FOx re-challenge in 1 patient (3.4%); gemcitabine/nab-paclitaxel association in 8 patients (27.5%); intra-arterial chemotherapy in 1 patient (3.4%). Two patients (6.8%) received a third line treatment: gemcitabine in 1 patient (3.4%); capecitabine in 1 patient (3.4%).

All evaluable patients with an increased Ca19.9 baseline value had a >20% decrease: 58% ≥50% decrease, 42% ≥70% and 90% decrease. CA19-9 levels were not significantly correlated with PFS and OS.

### Dose-intensity

Median number of administered cycles was 2 (range 1-11).

Median received dose intensities (rDI) per cycle were: 5-FU 1268.5 (375-1800) mg/m^2^/w, 70.4% of projected-DI (pDI); CPT-11 56 (30-80) mg/m^2^/w, 70%; OXP 29 (11-40) mg/m^2^/w, 72.5% (Table 3). Median rDI per patient were: 5-FU 1484.25 (375-1800) mg/m^2^/w, 82.4% of pDI; CPT-11 63.25 (30-80) mg/m^2^/w, 79%; OXP 33.5 (0-40) mg/m^2^/w, 83.75%. In yE patients, median rDIs per cycle were: 5-FU 1500 (375-1800) mg/m^2^/w, 83.3% of pDI; CPT-11 64 (30-80) mg/m^2^/w, 80%; OXP 34 (11-40) mg/m^2^/w, 85%.

**Table 3:** Dose-intensity

		All patients		Young-elderly patients	
		DI/cycle mg/m^2^/w		DI/cycle mg/m^2^/w	
	Projected DI mg/m^2^/w	Median (Range)	Received DI (%)	Median (Range)	Received DI (%)
**5-FU**	1800	1268.5 (375-1800)	70.4	1500 (375-1800)	83.3
**CPT-11**	80	56 (30-80)	70	64 (30-80)	80
**OXP**	40	29 (11-40)	72.5	34 (11-40)	85

Abbreviations: DI, dose-intensity; 5-FU, 5-fluorouracil; CPT-11, irinotecan; OXP, oxaliplatin.

### Toxicity

Table 4 describes cumulative toxicities in 29 enrolled patients, and 100 administered cycles. Cumulative G3-5 toxicities, by patients, were: diarrhea 5 patients (17%), stomatitis/mucositis 2 (6%), asthenia 4 (14%), nausea 1 (3%), vomiting 1 (3%), hypoalbuminemia 1 (3%), hypokalaemia 2 (7%), hypertransaminasemia 2 (7%), hyperbilirubinemia 1 (3%), hypercreatininemia 1 (3%), anemia 1 (3%), neutropenia 5 (17%), thrombocytopenia 1 (3%). The prevalent limiting toxicities (LT) were diarrhea, asthenia, neurotoxicity, thrombocytopenia. Cumulative G2 toxicities, by patients, were: nausea 10 (34%), vomiting 2 (7%), diarrhea 9 (31%), stomatitis/mucositis 4 (14%), hypoalbuminemia 2 (7%), asthenia 10 (34%), neurotoxicity 2 (7%), hypokalaemia 1 (3%), hypertransaminasemia 4 (14%), hyperbilirubinemia 1 (3%), anemia 3 (10%), neutropenia 6 (21%), thrombocytopenia 1 (3%). One case of toxic death (3%), due to G5 diarrhea, G4 mucositis, G4 thrombocytopenia, G3 anemia, associated to G3 hypoalbuminemia, G3 hypokaliemia, G3 hypercreatinemia, G3 neutropenia, and G2 asthenia, was observed. Five out of 29 patients (17%) discontinued FIr/FOx treatment due to limiting toxicity (neurotoxicity in 2 patients, asthenia in 1, thrombocytopenia in 1, toxic death in 1).

**Table 4:** Cumulative toxicity

	Patients					Cycles				
*Number*	29					100				
*NCI-CTC Grade*	1	2	3	4	5	1	2	3	4	5
Nausea (%)	5 (17)	10 (34)	1 (3)	-	-	31 (31)	13 (13)	1 (1)	-	-
Vomiting (%)	10 (34)	2 (7)	1 (3)	-	-	15 (15)	3 (3)	1 (1)	-	-
Anorexia (%)	10 (34)	1 (3)	1 (3)	-	-	15 (15)	3 (3)	1 (1)	-	-
Diarrhea (%)	5 (17)	9 (31)	4 (14)	-	1 (3)	38 (20.5)	14 (18)	4 (15)	-	1 (1)
Hypoalbuminemia (%)	-	2 (7)	1 (3)	-	-	-	2 (2)	1 (1)	-	-
Constipation (%)	7 (24)	7 (24)	1 (3)	-	-	11 (11)	7 (7)	1 (1)	-	-
Stomatitis/mucositis (%)	7 (24)	4 (14)	1 (3)	1 (3)	-	16 (16)	5 (5)	1 (1)	1 (1)	-
Erythema (%)	1 (3)	-	-	-	-	1 (1)	-	-	-	-
Asthenia (%)	10 (34)	10 (34)	4 (14)	-	-	64 (64)	17 (17)	4 (4)	-	-
Neurotoxicity (%)	15 (52)	2 (7)	-	-	-	61 (61)	4 (4)	-	-	-
Hypertension (%)	1 (3)	-	-	-	-	2 (2)	-	-	-	-
Hypotension (%)	-	-	-	-	-	-	-	-	-	-
Gengivitis (%)	-	-	-	-	-	-	-	-	-	-
Rhinitis (%)	3 (10)	-	-	-	-	3 (3)	-	-	-	-
Epistaxis (%)	4 (14)	-	-	-	-	4 (4)	-	-	-	-
HFS (%)	-	-	-	-	-	-	-	-	-	-
Hyponatriemia (%)	1 (3)	-	-	-	-	1 (1)	-	-	-	-
Hypokalemia (%)	1 (3)	1 (3)	2 (7)	-	-	1 (1)	2 (2)	2 (2)	-	-
Hypertransaminasemy (%)	7 (24)	4 (14)	2 (7)	-	-	24 (24)	6 (6)	2 (2)	-	-
Hyperpigmentation (%)	-	-	-	-	-	-	-	-	-	-
Fever without infection (%)	2 (7)	-	-	-	-	2 (2)	-	-	-	-
Alopecia (%)	3 (10)	5 (17)	1 (3)	-	-	8 (8)	8 (8)	6 (6)	-	-
Hyperbilirubinemia (%)	2 (7)	1 (3)	1 (3)	-	-	2 (2)	1 (1)	1 (1)	-	-
Hypercreatininemia (%)	-	-	1 (3)	-	-	-	-	1 (1)	-	-
Anemia (%)	5 (17)	3 (10)	1 (3)	-	-	13 (13)	4 (4)	1 (1)	-	-
Leucopenia (%)	3 (10)	3 (10)	4 (14)	-	-	4 (4)	7 (7)	5 (5)	-	-
Neutropenia (%)	-	6 (21)	5 (17)	-	-	-	13 (13)	9 (9)	-	-
Thrombocytopenia (%)	1 (3)	1 (3)	-	1 (3)	-	5 (5)	1 (1)	-	1 (1)	-

Abbreviations: NCI-CTC, National Cancer Institute Common Toxicity Criteria.

Overall, LTS were observed in 8 patients (27.5%) (Table 5), 5 out of 13 yE/oE patients (38.1%): 1 (3.4%) LTS-ss, and 7 (24.1%) LTS-ms. LTS-ms, consisting of a LT associated to other, at least G2, non-limiting toxicities were detected in 6 patients (20.6%); ≥ 2 LTs in 1 patient (3.4%). LTS were not significantly represented by LTS-ms compared to LTS-ss. The 1 LTS-ss was characterized by G3 diarrhea.

**Table 5:** Limiting Toxicity Syndromes (LTS): overall and in elderly patients

	Overall		Elderly	
	N.	%	N.	%
**Patients**	29	100	13	100
**Limiting Toxicity Syndromes (LTS)**	8	27.5	5	38.4
**LTS single-site (LTS-ss)**	1	3.4	-	-
**LTS multiple-sites (LTS-ms)**	7	24.1	5	38.4
Single LT plus G2-3	6	20.6	4	30.7
Double LTs	1	3.4	1	7.6

Abbreviations: LT, limiting toxicity; G, grade.

The 6 LTS-ms, consisting of LT associated to other, at least G2, non-limiting toxicities, were characterized by (Table 6): G2 neurotoxicity associated with G2 nausea, G2 vomiting, G2 diarrhea, G2 asthenia, G2 neutropenia; G2 thrombocytopenia associated with G2 asthenia, G3 leuconeutropenia, G2 ipokaliemia, G2 hypoalbuminemia, G2 hypertansaminasemia, G2 asthenia, G2 anorexia; G2 thrombocytopenia associated with G2 diarrhea, G2 neutropenia, G2 alopecia, G2 hypertransaminasemia; G3 asthenia associated with G3 alopecia and G3 leuconeutropenia; G2 neurotoxicity associated with G2 nausea, G2 diarrhea, G2 constipation, G2 alopecia, G2 hypertransaminasemia, G3 neutropenia; G3 diarrhea associated with G2 nausea, G2 anorexia. LTS-ms, with double/more LTs, was reported in 1 patient (3.4%) and characterized by G5 diarrhea, G4 mucositis, G4 thrombocytopenia and G3 anemia associated with G2 asthenia, G3 hypoalbuminemia, G3 hypokaliemia, G3 hypercreatininemia, G3 leuconeutropenia.

**Table 6:** Limiting Toxicity Syndromes (LTS)

Patients #	Age (years)	LT	Associated Toxicity	
			LT	G2-G3
**4**	61	Diarrhea G3	-	-
**1**	63	Neurotoxicity G2	-	Nausea G2 Vomiting G2 Diarrhea G2 Asthenia G2 Neutropenia G2
6	73	Thrombocytopenia G2	-	Anemia G2 Leuconeutropenia G3 Ipokalemia G2 Hypoalbuminemia G2 Hypertransaminasemia G2 Asthenia G2 Anorexia G2
16	66	Thrombocytopenia G2	-	Diarrhea G2 Neutropenia G2 Alopecia G2 Hypertransaminasemia G2
23	76	Asthenia G3	-	Alopecia G3 Leuconeutropenia G3
26	53	Neurotoxicity G2	-	Nausea G2 Diarrhea G2 Constipation G2 Alopecia G2 Hypertransaminasemia G2 Neutropenia G3
28	72	Diarrhea G3	-	Nausea G2 Anorexia G2
20	68	Diarrhea G5	Mucositis G4 Thrombocytopenia G4 Anemia G3	Asthenia G2 Hypoalbuminemia G3 Hypokalemia G3 Hypercreatininemia G3 Leuconeutropenia G3

Abbreviations: LT, limiting toxicity; G, grade.

## DISCUSSION

Triplet chemotherapy according to FIr/FOx schedule met projected high activity as first-line treatment of metastatic PDAC patients, reaching the first step of activity according to Simon-two step design: ORR 50% in the intent-to-treat and 53% in the as-treated analysis, with PFS 4 months (10.3% of patients progression-free > 12 months), and OS 11 months (27.5% of patients alive > 12 months), in the preliminary analysis of efficacy. Activity and clinical outcome of FIr/FOx exceeded that reported with gemcitabine: median OS 5.7 months, and 1-year OS rate 20%, median PFS 2.08 months, ORR 5.4% [1, 2]. Activity and clinical outcome may be higher than those reported with first generation gemcitabine-based combinations, excluding nab-paclitaxel: ORR 6.9-26.8%, median PFS 2.7-6 months, median OS 5.7-9 months [5–16].

Recently, phase III trials evaluating more intensive first-line chemotherapy regimen, such as gemcitabine plus nab-paclitaxel and triplet FOLFIRINOX, demonstrated to be much more, and equivalently effective, with significantly increased survival benefit over standard gemcitabine alone in metastatic PDAC patients [24]: ORR 23% and 31.6%, median PFS 5.5 and 6.4 months, OS 8.7 and 11.1 months, respectively. In the FOLFIRINOX study, median OS was significantly prolonged up to 11.1 months, with an increase of 4.3 months, compared with 6.8 months in the gemcitabine arm (hazard ratio for death, 0.57; *P* < 0.001) [24]. OS rate at 12 months was 48.4%, compared with 20.6% in the gemcitabine arm. In the recently reported phase III trial proposing gemcitabine and nab-paclitaxel association, 12-months OS rate was 35% [23]. Activity and clinical data reported with FIr/FOx in the present study are in the range of those reported with conventional intensive first-line treatment in PDAC patients. Thus, more active first-line treatment of metastatic PDAC can contribute to increase efficacy. FIr/FOx schedule may increase activity and efficacy of metastatic PDAC, with clinical outcome overlapping that reported with other triplet chemotherapy schedules, and evaluated in phase III randomized trials, as previously reported in MCRC setting [26, 27].

Our present real life study on consecutive, unselected patients showed that 13 patients (44.8%) were not evaluable in the ITT analysis because they did not received at least 3 cycles of treatment, thus confiming that, even today, the primary challenge of clinical management of metastatic PDAC patients is to start and safely perform at least 3 cycles of intensive chemotherapy treatment, to evaluate activity contributing to increase clinical outcome.

Among patients treated with intensive triplet FIr/FOx regimen, PFS and OS were not significantly different among patients treated with modulated and standard drug dosage, due to clinical parameters requiring treatment modulations. PS 2 significantly affected worse OS (1 compared with 12 months, *P* = 0.022), thus confirming overall benefit in clinical outcome achieved by metastatic PDAC patients with PS 0-1, treated with gemcitabine-based combinations [17]. In the MPACT trial, PS, presence of liver metastases, age, and number of metastatic sites involved were independent prognostic factors for OS and PFS [39, 40]. In our present study, PFS and OS seemed not significantly different according to primary tumor location (head or not), nor according to liver or other metastatic site, even if the small number of enrolled patients limited the relevance of subgroup analyses.

Median rDIs were >80% of the projected dose for each drug, also in elderly patients. Cumulative G3-5 toxicities were prevalently represented by: diarrhea (17%), stomatitis/mucositis (6%), asthenia (14%), nausea (3%), vomiting (3%), hypoalbuminemia (3%), hypokalaemia (7%), hypertransaminasemia (7%), hyperbilirubinemia (3%), hypercreatininemia (3%), anemia (3%), neutropenia (17%), thrombocytopenia (3%). In the previously reported phase II trial proposing intensive first-line triplet chemotherapy plus bevacizumab according to FIr-B/FOx regimen, as first-line treatment in MCRC patients, cumulative G3-4 toxicities were similar: diarrhea (28%), stomatitis/mucositis (6%), asthenia (6%), hypertension (2%), hypertransaminasemy (4%), neutropenia (10%). Triplet FIr/FOx, even associated to bevacizumab, determined only 10% G3-4 neutropenia, while FOLFOXIRI schedule, added or not to bevacizumab [26, 27], prevalently induced it (50%, equivalently) and also febrile neutropenia (6% and 8.8%, respectively) [30, 31]. In the phase III trial proposing FOLFIRINOX [24] (OXP 85 mg/m^2^, CPT-11 180 mg/m^2^, leucovorin 400 mg/m^2^, and 5-FU 400 mg/m^2^ as bolus followed by 2400 mg/m^2^ as 46-hour continuous infusion, every 2 weeks), the safety profile was less favourable than that reported in the gemcitabine arm [25]. More adverse events were reported in the FOLFIRINOX group: febrile neutropenia 5.4%; grade 3-4 neutropenia 45.7%, thrombocytopenia 9.1%, diarrhea 12.7%, and sensory neuropathy 9%. Filgrastim was administered in 42.5% of patients who received FOLFIRINOX. The intensive biweekly schedule, addiction of leucovorin to 5-FU, bolus 5-FU administration, could explain the less favourable haematological toxicity profile, particularly in term of neutropenia and febrile neutropenia.

In the phase III trial, gemcitabine 1000 mg/m^2^ plus nab-paclitaxel 125 mg/m^2^ association, 3 out of 4 weeks [23], prevalent G3-4 adverse events were: neutropenia (38%), febrile neutropenia (3%), thrombocytopenia (13%), anemia (13%), asthenia (17%), neurotoxicity (17%), diarrhea (6%). Granulocyte colony stimulating factor was administered in 26% of patients who received gemcitabine plus nab-paclitaxel. Dose modulations and treatment delays guaranteed more safely administration of gemcitabine and nab-paclitaxel association, and not significantly affected efficacy [40].

In the present study, LTS were observed in 27.5% of individual patients and in 38.4% of elderly patients treated with FIr/FOx regimen. The innovative clinical evaluation of LTS, consisting of at least the LT associated or not to other G2 or LT, introduced to better evaluate, in the individual patient, the presence of LT alone, LTS-ss, or the association of major toxicities in different sites, LTS-ms, showed that: overall, they were 3.4% and 24.1%, respectively; among elderly patients, they were all LTS-ms 38.4%. LTS were not significantly represented by LTS-ms compared to LTS-ss, even if the small number of enrolled patients requires further analyses. LTS-ms were mostly represented by diarrhea, mucositis, asthenia, neurotoxicity, thrombocytopenia and/or anemia, associated to nausea, vomiting, anorexia and/or neutropenia, hypokaliemia, hypoalbuminemia, hypertransaminasemia. In the individual patient, limiting and moderate toxicities often characterized LTS, previously observed in 44% MCRC patients treated with FIr-B/FOx, and equally involving single or multiple sites [27, 32].

Pharmacogenomic analysis evaluating 5-FU degradation rate (FUDR) and/or detection of a panel of DNA Single Nucleotide Polimorphisms (SNPs) involving different genes, such as *DPYD*, *UGT1A1*, *ABCB1*, *CYP3A4*, specifically influencing fluoropyrimidines and CPT-11-related adverse events, justifying inter-patients variability in safety profile, may help selection of patients fit for triplet chemotherapy, and may predict the occurrence of individual LTS, prevalently gastrointestinal [34–36, 41, 42]. Their predictive role should be prospectively verified, to be used in clinical practice.

Reported data confirmed that intensive regimens, such as FIr/FOx, frequently required proper clinical management of toxicity and treatment modulations due to moderate/severe toxicities. Careful selection of eligible patients, based on age, PS, comorbidity index, and monitoring of individual safety, also according to LTS in individual patients, are major parameters to optimize clinical management of metastatic PDAC. More, close monitoring of patients, expertise with a particular regimen, and toxicity management, remained the physician-related factors, that can guide personalized selection of first-line regimens in individual PDAC patients.

## MATERIALS AND METHODS

### Patient eligibility

Patients were eligible if they had clinical and/or histological/cytological confirmed diagnosis of measurable metastatic PDAC; age ≥18 years, specifically <65 years (non-elderly), ≥65 <75 years (yE), and ≥75 years (oE); WHO PS ≤ 2; adequate hematological, renal and hepatic functions; life expectancy more than 3 months.

Ineligibility criteria: pregnancy and breast-feeding; uncontrolled severe diseases; cardiovascular disease (uncontrolled hypertension, uncontrolled arrhythmia, ischemic cardiac diseases in the last year); thromboembolic disease, coagulopathy, pre-existing bleeding diatheses; sensory and/or motor polineuropathy; surgery within the previous 28 days; previous adjuvant chemotherapy or radiotherapy completed less than 6 months before. CIRS was used to evaluate the comorbidity status [37]. Primary CIRS stage consisted of: independent Instrumental Activity of Daily Living (IADL), and absent or mild grade comorbidities; intermediate CIRS stage consisted of dependent or independent IADL, and less than 3 mild or moderate grade comorbidities; secondary CIRS stage consisted of more than 3 comorbidities or a severe comorbidity, with or without dependent IADL.

Treatment was approved by Agenzia Italiana del Farmaco (AIFA) for administration *in label* for metastatic PDAC treatment in Italian public hospitals, and published in Gazzetta Ufficiale Repubblica Italiana (“Elenco dei Medicinali erogabili a totale carico del Servizio Sanitario Nazionale”, Gazzetta Ufficiale Repubblica Italiana N.1, 2 Gennaio 2009). The study was approved by the Regional Review Board (Regione Abruzzo, Italia, according to D.G.R. n.489, 25/05/2007), and conducted in accordance with the Declaration of Helsinki. All patients provided written, informed consent.

### Methods

#### Schedule

This was a single-arm phase II study evaluating safety and activity of weekly alternating 5-FU, CPT-11, and OXP (FIr/FOx) as first-line treatment of metastatic PDAC.

FIr/FOx association consisted of 5-FU associated to alternating CPT-11 or OXP according to the following weekly schedule: TFI/5-FU (Fluorouracil Teva; Teva Italia, Milan, Italy), 750-800-900 mg/m^2^/die, over 12-hour (from 10:00 p.m to 10:00 a.m.), days 1-2, 8-9, 15-16 and 22-23; CPT-11 (Campto; Pfizer, Latina, Italy), 120-140-160 mg/m^2^, administered over 90 minutes as an intravenous infusion in 250 ml of NaCl 0.9%, days 1 and 15; OXP (Eloxatin; Sanofi-Aventis, Milan, Italy) over 2-hours as an intravenous infusion in 250 ml of dextrose 5%, at the dose of 70-80 mg/m^2^, days 8 and 22. Cycles were repeated every 4 weeks. 5-FU was administered by a portable pump (CADD Plus, SEVIT) using a venous access device. According to patients’ fitness, and particularly in patients with PS 2, and/or ≥75 years, secondary CIRS stage, and/or abnormal liver functional laboratory tests, such as ≥ G2 hypertransaminasemia at baseline, drugs’ doses were modulated in individual patients as reported, providing a received DI >75% for each drug, reported as active and efficacious in previous studies of triplet chemotherapy regimens [24, 26–31].

#### Study design

Physical examination and routine laboratory studies were performed at baseline and every week on-treatment, including complete blood cell count, electrolytes, liver and renal function tests, urine examination and coagulation function; tumor markers every cycle; electrocardiogram every cycle, and echocardiogram at baseline, and every 3 cycles.

Primary end-point was ORR; secondary end-points were toxicity, PFS, OS. ORR was evaluated according to RECIST criteria [43]; PFS and OS using Kaplan and Meier method [44]. PFS was defined as length of time between the beginning of treatment and disease progression or death (resulting from any cause) or to last contact; OS as length of time between the beginning of treatment and death or to last contact. The log-rank test was used to compare PFS and OS [45]. Clinical evaluation of response was made by computerized tomography (CT)-scan; magnetic resonance imaging (MRI) and/or positron emission tomography (PET) were added based on the investigators’ assessment; objective responses were confirmed three months later. Follow-up was scheduled every three months, up to disease progression or death. Toxicity was monitored every week according to National Cancer Institute Common Toxicity Criteria (NCI-CTC, version 4.0). LT was defined as grade 3-4 non-haematological toxicity (mainly represented by diarrhea, mucositis, neurotoxicity, hand-foot syndrome, asthenia, liver functional tests), grade 4 hematologic toxicity, G4 neutropenia, febrile neutropenia, G3-4 thrombocytopenia, or associated with significant clinical bleeding, grade 3-4 anemia, G2-3 neurotoxicity, or any toxicity determining a > 2 weeks treatment delay.

LTS, consisting of at least a LT associated or not to other limiting or G2 toxicities, were evaluated as previously reported [27, 32]. These were classified as: LTS-ss, if characterized only by the LT; LTS-ms, if characterized by ≥ 2 LTs or a LT associated to other, at least G2, non-limiting toxicities. Chi-square test was used to compared the rates of LTS-ms and LTS-ss [46].

Correlations between maximum decrease from baseline in CA19.9 level and PFS and OS were analyzed, to assess possible relationships between CA19.9 and clinical outcomes.

#### Statistical design

This phase II study was planned according to two-steps Simon’s design [38]: assuming as minimal interesting activity an ORR 10%, 1 objective response among the first 10 enrolled patients was necessary for the first-step; to verify the alternative hypothesis of ORR 30%, 5 objective responses among the total 29 enrolled patients were necessary; power (1 - β) 80%; error probability α 5%. p_0_ was considered as the estimated activity reported with gemcitabine alone (median ORR 10%), and confirmed with the association of gemcitabine plus erlotinib (ORR 8.6%) [1–5, 16]; p_1_ as the projected ORR using the present intensive triplet combination, according to FIr/FOx schedule, increasing the activity ≥ 20% in metastatic PDAC patients, as reported with FOLFIRINOX (ORR 31.6%), and with the association of gemcitabine and nab-paclitaxel in the phase I/II trial (ORR 46% in the overall population, and 48% in patients treated at the recommended dose of nab-paclitaxel 125 mg/m^2^; ORR 23% in the more recently reported phase III trial) [22–24].

## CONCLUSIONS

FIr/FOx intensive triplet chemotherapy in metastatic PDAC patients preliminary showed high activity. Present schedule was feasible in non-elderly and elderly patients, with PS 0-1, with manageable toxicities, at proper CPT-11, OXP, and 5-FU doses. LTS were prevalently characterized by diarrhea, mucositis, asthenia, anemia, neurotoxicity and/or thrombocytopenia, associated to nausea, vomiting, anorexia and/or neutropenia. Elderly patients preliminary showed trendy, but not significantly worse OS. Adequate selection of suitable patients, based on clinical parameters, aimed to maintain safety profile at efficacious DIs, will verify if more intensive approaches, such as triplet chemotherapy regimen could increase OS, compared to historical gemcitabine control, in the clinical practice management of metastatic PDAC patients, and if it could be a treatment option in locally advanced/borderline resectable pancreatic cancer patients.

## Abbreviations

CIRS: Cumulative Illness Rating Scale
CPT-11: irinotecan
DI: dose intensity
IADL: Instrumental Activity of Daily Living
LT: limiting toxicity
LTS: limiting toxicity syndromes
LTS-ms: limiting toxicity syndromes multiple sites
LTS-ss: limiting toxicity syndromes single site
MCRC: metastatic colorectal cancer
oE: old-elderly
OR: objective response
ORR: objective response rate
OS: overall survival
OXP: oxaliplatin
PDAC: pancreatic ductal adenocarcinoma
pDI: projected dose intensity
PFS: progression-free survival
PS: performance status
rDI: received dose intensity
TFI: timed-flat-infusion
yE: young-elderly
WHO: World Health Organization
5-FU: 5-fluorouracil
